The article "Reexamining the effects of electrode location on measures of neural health in cochlear implant users" was published in 2023. Journal: JASA Express Lett.

# Reexamining the effects of electrode location on measures of neural health in cochlear implant users

**DOI:** 10.1121/10.0019806

**Published:** 2023-06-26

**Authors:** Kara C. Schvartz-Leyzac, Bryan E. Pfingst

**Affiliations:** 1 Medical University of South Carolina, Department of Otolaryngology-Head & Neck Surgery, 135 Rutledge Avenue, Charleston, South Carolina 29425, USA; 2 University of Michigan, Kresge Hearing Research Institute, Department of Otolaryngology- Head & Neck Surgery, 4605 Medical Science Unit II, Ann Arbor, Michigan 48109, USA leyzac@musc.edu, bpfingst@umich.edu

## Abstract

The electrically evoked compound action potentials (ECAPs) amplitude-growth function (AGF) slope correlates with spiral ganglion neuron (SGN) density in the cochlear implanted cochlea. Electrode insertion angle and medial–lateral distance covary from base to apex; in some human ears, SGN survival varies from base to apex, making it difficult to parse out contributing factors to the ECAP AGF slope. Evoked compound action potentials were analyzed on each electrode and compared to post-operative computerized tomography scans. When controlling for medial–lateral distance, insertion angle does not influence ECAP AGF slope.

## 1. Introduction

Cochlear implants (CIs) often provide significantly improved speech understanding to recipients of all ages, yet outcomes vary widely across patients. Emerging data suggest that the condition of the auditory nerve [i.e., spiral ganglion neuron (SGN) density] influences speech recognition outcomes (Kamakura and Nadol, 2016; Schvartz-Leyzac and Pfingst, 2018). Using animal models of cochlear implantation, studies have shown that objective measures, such as the electrically evoked compound action potential (ECAP) are correlated with the density of remaining spiral ganglion neurons (SGNs) (Prado-Guitierrez *et al.*, 2006; Ramekers *et al.*, 2014; Ramekers *et al.*, 2015; Schvartz-Leyzac *et al.*, 2020a). Specifically, these studies reveal that suprathreshold ECAP measures account for approximately 40%–60% of the residual SGN density in cochlear implanted animals.

These same ECAP measures have been shown to sometimes relate to speech recognition outcomes in CI users (van Eijl *et al.*, 2017). Scheperle (2017) reported that the across-site average of the peak amplitude of the ECAP amplitude-growth function (AGF) was correlated with post-operative measures of vowel recognition in adult CI recipients (Scheperle, 2017); DeVries *et al.* (2016) reported a similar relationship. Schvartz-Leyzac and Pfingst (2018) showed that, among bilaterally implanted CI recipients, larger across-site mean interphase gap (IPG) effect for ECAP amplitudes and AGF slopes were observed in the ear with better speech understanding in noise within each subject (Schvartz-Leyzac and Pfingst, 2018). The IPG effect is the change in a given ECAP metric (e.g., amplitude or AGF slope) caused by increasing the IPG between the first and second phase of the biphasic pulse (Ramekers *et al.*, 2014; Schvartz-Leyzac *et al.*, 2020a). While the relationship between ECAP measures and speech recognition outcomes has varied across studies, several studies support a link between these two variables. Some studies have also shown that the ECAP amplitude and AGF slopes vary depending on electrode location within the cochlea, sometimes with larger amplitudes and AGF slopes present in the apical compared to basal electrodes (Brill *et al.*, 2009; van de Heyning *et al.*, 2016). Conversely, there is no consistent basal-to-apical trend for the IPG effect for ECAP amplitude and AGF slope (Schvartz-Leyzac and Pfingst, 2016; Schvartz-Leyzac *et al.*, 2020b).

The article "Reexamining the effects of electrode location on measures of neural health in cochlear implant users" was published in 2023. Journal: JASA Express Lett.

Electrode location also influences ECAP measures in CI recipients. Medial–lateral distance of the electrode, for example, influences some ECAP measures in animals (cats) and humans (Shepherd *et al.*, 1993; Schvartz-Leyzac *et al.*, 2020b). Medial–lateral distance can be defined as the distance between the electrode contact and the cochlear medial wall (MW) or the mid-modiolar axis (MMA) and the distinction is important, given that the location and morphology (e.g., presence/absence of dendrites) of the surviving SGNs is unknown for each subject. Furthermore, the site of excitation along the SGN population is also not necessarily known, given the largely uncontrolled current flow within the cochlea. Based on these factors, the precise site of excitation is not easy to predict. Results described in Schvartz-Leyzac *et al.*, 2020 suggest that threshold and suprathreshold ECAP measures are related to the distance between the electrode and MMA, but not necessarily the MW (Schvartz-Leyzac *et al.*, 2020b), suggesting a more central site of excitation. These previous studies did not afford the opportunity to examine the influence of other electrode placement factors, such as scalar location, due to the limited sample size.

Post-mortem temporal bone studies in humans reveal that, among patients with sensorineural hearing loss, the pattern of residual SGNs varies from base to apex in the cochlea—sometimes with fewer SGNs remaining in the basal portion, compared to medial and apical turns (Hinojosa and Marion, 1983; Nadol, 1997). Coupled with other findings showing covariance of medial–lateral distance with insertion angle (Schvartz-Leyzac *et al.*, 2020b), it could be inferred that ECAP amplitude and slope measured with a fixed IPG is related to residual SGNs, medial–lateral distance, or both of these factors. For instance, a lower ECAP AGF slope value on a basal electrode could be due to poorer SGN survival, greater medial–lateral distance, or a combination of these factors.

The article "Reexamining the effects of electrode location on measures of neural health in cochlear implant users" was published in 2023. Journal: JASA Express Lett.

Understanding and characterizing the impact of electrode placement on functional measures of cochlear health, such as the ECAP, is important to better use such measures in a clinical application. The present study is an extension of previous work (Schvartz-Leyzac *et al.*, 2020b) examining effects of electrode location on ECAP measures in an expanded group of CI participants. The overarching goal is to more precisely describe individual contributions of covarying factors, such as basal-to-apical location, medial–lateral distance, and scalar location, to ECAP measures in CI recipients.

## 2. Methods

### 2.1 Participants

Participants included 11 CI recipients previously reported in Schvartz-Leyzac *et al.* (2020b), in addition to 13 additional CI recipients (male = 8; ages 44–80 years), who participated since that time; one of these additional 13 participants was bilaterally implanted and data were collected in both ears. Therefore, 25 implanted ears were evaluated for the current study. Demographic information from the initial 11 participants can be found in Schvartz-Leyzac *et al.* (2020b). Ears added to the new analysis (N = 14) included adult recipients of Cochlear™ implant systems (Centennial, CO) [CI612 (perimodiolar) or CI622 (straight/lateral)] electrode arrays, who had at least 6 months of CI experience. Table 1 provides demographic information for the 14 ears added to the new analysis.

**Table 1.** Demographic information for new participants (those not included in Schvartz-Leyzac *et al.*, 2020b).^a^^,^^b^

Participant ID	Sex	Age	Onset of hearing loss	Etiology	Ear	Years of implant use	Device
CI01L	M^a^	58	Teenager	Hereditary	L^c^	1.5	CI612
CI01R					R^d^	2	CI612
CI02	M	73	65 years of age	Unknown	R	1	CI622
CI03	M	72	40 years of age	Noise exposure	R	1.5	CI622
CI04	M	42	8 years of age	Infection	R	1	CI612
CI05	F	49	Teenager	Unknown	R	1.5	CI612
CI06	F	67	9 years of age	Ototoxicity	R	0.6	CI622
CI07	M	62	30–39 years of age	Noise exposure	L	1	CI612
CI09	M	79	50–59 years of age	Unknown	L	1.5	CI622
CI10	M	47	43	Noise exposure	R	0.6	CI612
CI11	F	61	55	Unknown	R	0.6	CI622
CI12	F	45	30–39 years of age	Hereditary	R	1	CI612
CI13	F	61	40–49 years of age	Unknown	L	0.6	CI622
CI14	M	71	11 years of age	Meniere's disease	R	3.5	CI512

^a^ M, male.

^b^ F, female.

^c^ L, left.

^d^ R, right.

### 2.2 Electrically evoked compound action potentials (ECAPs)

ECAPs were measured on all available electrodes in each ear, using the forward-masking artifact reduction method (Abbas *et al.*, 1999; Abbas *et al.*, 2004). ECAPs were not measured on electrodes deactivated in the participant's clinical program, and could not always be measured due to recording artifact, poor morphology, limited dynamic range, or compliance issues (9% of electrodes). ECAPs were collected using Cochlear Corporation CustomSound EP Version 6.0 or later, using neural response telemetry (NRT), and methods for collection were identical to those described in Schvartz-Leyzac *et al.* (2020). Default parameters were used for most participants (80 pps stimulation rate, 20 kHz sampling rate, 50–100 sweeps per average). The recording delay (default = 122 *μ*s) and gain (50 dB) were sometimes adjusted to improve morphology. Before measuring ECAPs on each electrode, the maximum tolerable stimulation level was determined on each electrode for each condition to ensure that all stimuli were comfortable.

The article "Reexamining the effects of electrode location on measures of neural health in cochlear implant users" was published in 2023. Journal: JASA Express Lett.

We measured the ECAP AGF on each electrode, with current levels ranging from just below ECAP threshold to the maximum tolerable stimulation level. The current level step size was 5 clinical units (CUs). Current units are expressing in *μ*A below equation, where CU represents clinical units specified in the Cochlear software:

$$(\;\mu A=17.5\;*100^{\wedge }(CU/255).$$

For each recording, the peak-to-peak ECAP amplitudes were measured from the leading negative peak (N1) to the following positive peak (P2) using the CustomSound**^®^** EP software. The AGF for each electrode was measured 2–3 times for each condition (seven and 30 *μ*s IPGs, as outlined below). At least four data points were required to fit the slope function (dynamic range = 15 CU). Approximately 9% of the electrodes evaluated used only four data points to fit the AGF, while the maximum number of data points in an AGF was 15. We obtained amplitude-growth functions (AGFs) on each electrode for two IPG durations of 7 and 30 *μ*s. Otherwise, parameters were identical to those described in previous studies (Schvartz-Leyzac and Pfingst, 2016, 2018).

ECAP AGF slopes (*μ*V/*μ*A) (converted from CUs) were fit using methods consistent with previous studies (Schvartz-Leyzac *et al.*, 2020a; Schvartz-Leyzac *et al.*, 2021; Skidmore *et al.*, 2022) and are briefly described here. All points below 5 *μ*V (noise floor) were excluded (noise floor level available from the manufacturer). The AGF was linearized by approximating the slope of the linear region using the “gradient” function in matlab, and systematically removing the points that deviated by more than 20% of this slope. A linear model *(y = y0 +ax)* was fit to all of the remaining points and the resulting slope was calculated. In all cases, the linear fit was statistically significant and produced an R^2^ of 0.95 or higher. The change (increase or decrease) in slope or threshold as a function of the IPG (the “IPG Effect”) was also calculated for each electrode by subtracting the fitted AGF slope for the 7 *μ*s IPG stimulus from that for the 30 *μ*s IPG stimulus.

The article "Reexamining the effects of electrode location on measures of neural health in cochlear implant users" was published in 2023. Journal: JASA Express Lett.

### 2.3 Post-operative computerized tomography (CT)

Post-operative imaging was completed using advanced CT methods to better assess the position of the electrode array within the cochlea. The CT methods used here are more detailed than standard clinical CT methods. For the 11 participants previously reported on in Schvartz-Leyzac *et al.* (2020), CT methods were previously described and were consistent with previous studies as well (Skinner *et al.*, 2007; Teymouri *et al.*, 2011; Long *et al.*, 2014; DeVries *et al.*, 2016). These data were collected at the University of Michigan (UM). The additional 14 ears were measured and analyzed (new data) at the Medical University of South Carolina (MUSC) using alternative CT methods to assess electrode locations (Noble *et al.*, 2013; Noble *et al.*, 2014; Noble *et al.*, 2016; O'Connell *et al.*, 2016a; Zhang *et al.*, 2018). Different CT methods used at UM and MUSC were due to standard clinical care and/or research practices used at each institution. These methods have not been formally compared, but they derive similar electrode location characteristics, such as medial–lateral distance, scalar location, and insertion depth/angle. To make sure that CT analysis and testing location did not significantly influence results, statistical models described in Sec. 2.4 include CT analysis type as a covariate.

Post-operative CT metrics of interest included (1) medial–lateral distance, defined as the distance between the electrode and mid-modiolar axis (MMA), (2) insertion angle/depth, and (3) scalar location. Scalar location is dichotomously categorized into scala tympani or scala vestibuli. Intermediate locations that could not be precisely determined and were labeled as residing in an intermediate region (“M-region”) but were not included for analysis.

### 2.4 Statistical analysis

All data were analyzed using matlab (Natick, MA) and R Version 4.0.3 (Vienna, Austria) (R-CoreTeam, 2020). In keeping with previous studies and as described in Sec. 2.2, a custom fitting method was used to fit a linear function to the ECAP AGFs to derive a slope measure. Linear mixed models were constructed in R using lme4 (Bates *et al.*, 2015) and lmerTest (Kuznetsova *et al.*, 2017) and using random subject effects (1 | Subject) to determine the relationship between medial–lateral distance, insertion angle, and ECAP measures. Covariance factors were entered appropriately to determine (1) if variables of interest were affected by CT analysis type and (2) to evaluate the independent effects and interaction between CT metrics (insertion angle, medial–lateral distance, and scalar location) on the ECAP AGF linear slope. Plots were examined and analyzed to ensure sure that statistical assumptions (linear relationship between independent and dependent variables, errors have constant variance, errors are independent, and errors are normally distributed), were not violated for analyses. The statistics for all fitted models are summarized in Table 2.

The article "Reexamining the effects of electrode location on measures of neural health in cochlear implant users" was published in 2023. Journal: JASA Express Lett.

**Table 2.** Statistics for linear mixed model analyses.

Effects	β	SE	t	df	p
Dependent variable: ECAP AGF Slope (7 *μ*s IPG)					
Medial–lateral distance	−0.157	0.021	−7.461	437.9	p < 0.001
Insertion angle	0.0009	0.0001	6.976	435.4	p <0.001
Scalar location	0.046	0.057	0.816	376.6	0.41
CT analysis method	−0.038	0.147	−0.263	25.0	0.79
Medial–lateral distance × CT analysis method	−0.021	0.042	−0.501	437.6	0.616
Insertion angle × CT analysis method	0.0004	0.0002	1.531	435.4	0.127
Scalar location × CT analysis method	0.058	0.116	0.507	377.0	0.613
Medial–lateral distance × Insertion angle	−0.0001	0.0001	−0.784	434.8	0.4333
Dependent variable: Medial–lateral distance (mm)					
Insertion angle	−0.0052	0.0001	−26.90	519.6	p < 0.001
Dependent variable: ECAP IPG effect					
Medial–lateral distance	−0.012	0.014	−0.833	425.5	0.402

## 3. Results

### 3.1 Relationship between medial–lateral distance and suprathreshold ECAP measures

The relationship between medial–lateral distance and the ECAP AGF slope for a fixed IPG of 7 *μ*s is shown in Fig. 1(A). Results showed a significant relationship between these two variables [t(437.98) = −7.461, p <0.001]. Specifically, the fitted model revealed that ECAP AGF slope decreased by an average 0.15 *μ*V/*μ*A (95% confidence intervals = −0.198 to −0.115) for every 1 mm increase in medial–lateral distance. It can also be observed that in four participants, the data show an opposite relationship (ECAP AGF slope increases with increasing distance). There is no obvious explanation why these four participants show a different result. In contrast to these results, no relationship was found between the IPG effect for the ECAP AGF linear slope and medial–lateral distance [t(425.56)= −0.833, p = 0.40], as shown in Fig. 1(B). These results are consistent with previous findings (Schvartz-Leyzac *et al.*, 2020b). As shown in Table 2, ECAP AGF slopes did not differ between the two testing sites (p = 0.79) (in Table 2, CT analysis method can be interpreted as a by proxy for test location).

The article "Reexamining the effects of electrode location on measures of neural health in cochlear implant users" was published in 2023. Journal: JASA Express Lett.

**Fig. 1.** Scatterplots showing the relationship between medial–lateral distance (mm) (*x* axis) and ECAP AGF linear slope (*μ*V/*μ*A) (A) or the IPG effect for ECAP AGF linear slope (*μ*V/*μ*A) (B). The light gray circles reflect individual data points for each participant and electrode contact on which the ECAP AGF slope was measured. The dark gray solid lines represent individual correlations (linear regression) between the *x*- and *y*-axis for each participant, and the solid thick black line represents the group level trend line.

### 3.2 Insertion angle and medial–lateral distance

Not surprisingly, the medial–lateral distance decreased as the insertion angle increased as shown in Fig. 2(A). A linear mixed effects model revealed that the medial–lateral distance decreased by 0.00527 mm (95% confidence intervals = −0.005 to 0.004) for every 1° increase in insertion angle [t(519.6) = 26.90, p < 0.001]. There was no significant interaction of array type (p > 0.05). Results also showed that the ECAP AGF slope increased as insertion angle increased. Specifically, the linear mixed effects model revealed that the slope increased by 0.009 *μ*V/*μ*A (95% CI = 0.0006–0.0012) for every 1° increase in insertion angle [t(435.4) = 6.976, p < 0.001)] [Fig. 2(B)]. This second finding is consistent with previous studies (Brill *et al.*, 2009; van de Heyning *et al.*, 2016).

**Fig. 2.** Scatterplots showing the relationship between insertion angle (*x* axis) and medial–lateral distance (A) or the ECAP AGF linear slope (B). The light gray circles reflect individual data points for each participant and electrode contact on which the ECAP AGF slope was measured.

The dark gray solid lines represent individual correlations (linear regression) between the *x*- and *y*- axis for each participant, and the solid thick black line represents the group level trend line.

### 3.3 Covariance of medial–lateral distance and insertion angle on ECAP measures

To better understand the relationship between covarying factors of medial–lateral distance and insertion angle on ECAP AGF slope, a linear mixed model analysis was performed by adding an interaction (covariance) between medial–lateral distance and insertion angle. As shown previously, ECAP AGF slope decreases with increasing medial–lateral distance [Fig. 1(A)] but increases with increasing insertion angle [Fig. 2(B)]. Medial–lateral distance decreases with increasing insertion angle [Fig. 2(A)]. Therefore, insertion angle was entered as a covarying factor with medial–lateral distance into a linear mixed model to assess the interaction between these variables (ECAP AGF linear slope = medial–lateral distance * insertion angle). Results are described in Table 2 and show that this model is non-significant [t(434.8) = −0.784, p = 0.43]. This means that the effect of medial–lateral distance on ECAP AGF slope values was not affected by the insertion angle. Therefore, the results suggest that, after accounting for effects of medial–lateral distance, insertion angle did not significant influence ECAP AGF slope.

The article "Reexamining the effects of electrode location on measures of neural health in cochlear implant users" was published in 2023. Journal: JASA Express Lett.

### 3.4 Effects of scalar location on ECAP AGF slope

The effects of scalar location on AGF slope are shown in Fig. 3. Due to the lack of precision, electrodes identified within the M-region were excluded from the analysis. A linear mixed model was constructed to better assess the effect of scalar location on ECAP AGF slope, and results are summarized in Table 2. As shown in Fig. 3, there was no significant difference between ECAP AGF slope values for electrodes located in the scala vestibuli vs the scala tympani [t(376.6) = 0.816, p = 0.41].

**Fig. 3.** Box plots comparing ECAP AGF linear slopes (*μ*A/*μ*V) between electrode contacts resolved within the scala tympani (darker gray) or scala vestibuli (lighter gray). Within each box plot, the horizontal black line/pinched area represents the median value within each group. The lower and upper limits to the box correspond to the first and third quartiles (the 25th and 75th percentiles). The lower and upper whisker extends from the 10th and 90th percentiles, respectively. The filled black symbols represent outliers.

### 3.5 Effect of CT analysis method and participant group

Although the two different CT analyses used in the present study produced similar metrics, additional models were constructed to determine whether there were significant differences in ECAP measures or CT variables across the two different groups of participants. Results are summarized in Table 2. A linear mixed model revealed that the ECAP AGF slopes did not significantly differ between participant group/CT analysis method [t(25) −0.263, p = 0.79]. Likewise, CT analysis was entered as a covariate for linear mixed model analysis to examine the relationships between ECAP AGF slope and medial–lateral distance, insertion angle, and scalar location. Similarly, there was no interaction between CT analysis method and medial–lateral distance (p = 0.61), insertion angle (p = 0.12), or scalar location (p = 0.61).

## 4. Discussion

Results presented here confirm previous findings using a larger sample size, and also extend those findings to better define underlying contributions to the ECAP AGF linear slope, which has been previously shown in animal models to reflect, at least in part, the condition of the auditory nerve in cochlear implanted ears (Ramekers *et al.*, 2014; Schvartz-Leyzac *et al.*, 2019; Schvartz-Leyzac *et al.*, 2020a). While there is the potential to use ECAP measures in humans to define neural health patterns across the electrode array and/or apply such measures to improve performance, it is important to better understand contributions of non-neural factors, such as electrode location. Of course, there are other non-neural factors that were not evaluated in the current study, such as impedance. Some of the difficulty in applying these measures in the clinical setting is that underlying factors of the ECAP AGF slope seem to covary. Previous animal studies that examined the relationship between ECAP AGF slope and underlying SGN density were performed under conditions of a highly constrained medial–lateral distance and insertion angle; this was due to the relatively larger size of the electrode array used compared to the smaller size of the guinea pig cochleae (Ramekers *et al.*, 2014; Pfingst *et al.*, 2017; Schvartz-Leyzac *et al.*, 2019; Schvartz-Leyzac *et al.*, 2020a). As shown here, in humans the insertion angle covaries with medial–lateral distance (Fig. 2) and the ECAP AGF slope increases with increasing insertion angle. Previous studies showing a similar trend have hypothesized that this relationship reflects increased SGN density in more apical regions (Brill *et al.*, 2009; van de Heyning *et al.*, 2016), and this assumption is also supported by post-mortem temporal bone studies citing some ears having relatively denser population of SGN fibers in the medial and apical portions compared to the base of the cochlea (Hinojosa and Marion, 1983; Nadol, 1997). However, medial–lateral distance also seems to be related to ECAP AGF measures (Schvartz-Leyzac *et al.*, 2020b and Fig. 1), making an overall interpretation of the data more difficult.

The article "Reexamining the effects of electrode location on measures of neural health in cochlear implant users" was published in 2023. Journal: JASA Express Lett.

Here, a statistical modeling approach was taken to better understand the covariance of these factors in a larger group of participants. Specifically, results showed a lack of significant covariance between independent variables, suggesting that medial–lateral distance and insertion angle are independently associated with ECAP AGF linear slopes (Table 2). These results suggest that, when controlling for medial–lateral distance, insertion angle does not influence ECAP AGF slope. Therefore, larger ECAP responses observed in the apex seem to be due to electrode location and are not strongly influenced by neural health.

Previous results also showed promising application of the IPG effect for ECAP AGF slope to improve speech recognition in CI users (Schvartz-Leyzac *et al.*, 2021) because this measure has been shown to also reflect SGN density in the implanted guinea pig (Ramekers *et al.*, 2014; Schvartz-Leyzac *et al.*, 2020a) but is not significantly influenced by medial–lateral distance (Schvartz-Leyzac *et al.*, 2020b). Results shown in Fig. 1(B) confirm previous findings that there is no correlation between the IPG effect for ECAP AGF slope and medial–lateral distance in a larger cohort of participants.

Last, electrode position can also be defined by the scalar location of each electrode contact. While scalar location has been shown to influence speech recognition outcomes (Finley *et al.*, 2008; Wanna *et al.*, 2014; O'Connell *et al.*, 2016b), its influence on ECAP measures had not yet been explored. Previous studies have shown that scalar location can vary widely within and across ears (Wanna *et al.*, 2014) with approximately 42% or 11% of electrode arrays translocating for perimodiolar or straight styles, respectively. Results described in the present study (Fig. 3, Table 2) show there was no significant difference in ECAP AGF slope values based on electrode scalar location. This graph also shows several outliers, which reveals that while the majority of participants had similar ECAP AGF slope values, there were some significantly larger slope values that were outliers, compared to the group mean. The important observation to note in Fig. 3 is that the outliers also seem to be fairly equal in number across the scala tympani and vestibuli, supporting the notion that scalar location has little effect on ECAP AGF slope. Although not certain, it is possible that at suprathreshold current levels used here, current spread is sufficiently broad that scalar location is not an influencing factor.

While the results described here are important, there is one important limitation that should be noted. The primary limitation of the current research is that data were analyzed using two comparable, but different, post-operative CT analyses. The details of both analyses are comprehensively explained elsewhere (Teymouri *et al.*, 2011; Noble *et al.*, 2013; Noble *et al.*, 2014; Noble *et al.*, 2016) for further reference, and both have been widely used across several CI studies. However, to date, there has been no direct comparison between the two approaches. While it is uncertain how the two methods compare directly, both methods are well validated using cadaver models and it is assumed, for the purpose of this study, that they can be comparably used. However, because this is not known directly, it remains a possible limitation of the study.

Overall, the results presented here offer further understanding of non-neural factors that contribute to the ECAP AGF slope measures, which has been shown to reflect the condition of the auditory nerve in the cochlear implanted ear. These results continue to suggest that, after accounting for medial–lateral distance, the ECAP slope using a fixed IPG does not vary from base to apex. This would suggest, at least in this cohort of ears, a lack of systematic variance in SGN density from base to apex.
